# The influence of a gene expression signature on the diagnosis and recommended treatment of melanocytic tumors by dermatopathologists

**DOI:** 10.1097/MD.0000000000004887

**Published:** 2016-10-07

**Authors:** Clay J. Cockerell, Jaime Tschen, Brent Evans, Emily Bess, John Kidd, Kathryn A. Kolquist, Colleen Rock, Loren E. Clarke

**Affiliations:** a Department of Dermatology and Pathology, University of Texas Southwestern Medical Center, Dallas; b St. Joseph Dermatopathology, Houston, TX; c Clinical Affairs; d Department of Dermatology; e Department of Histopathology, Myriad Genetic Laboratories, Inc., Salt Lake City, UT.

**Keywords:** clinical utility, melanoma, molecular diagnostic techniques, nevi and melanomas

## Abstract

It is well documented that histopathologic examination is sometimes inadequate for accurate and reproducible diagnosis of certain melanocytic neoplasms. Recently, a 23-gene expression signature has been clinically validated as an adjunctive diagnostic test to differentiate benign nevi from malignant melanomas. This study aimed to quantify the impact of this test on diagnosis and treatment recommendations made by dermatopathologists.

Diagnostically challenging melanocytic lesions encountered during routine dermatopathology practice were submitted for gene expression testing and received a melanoma diagnostic score (MDS). Submitting dermatopathologists completed a survey documenting pre-test diagnosis, level of diagnostic confidence, and recommendations for treatment. The survey was repeated after receiving the MDS. Changes between the pre- and post-test surveys were analyzed retrospectively.

When the MDS was available as part of a comprehensive case evaluation in diagnostically challenging cases, definitive diagnoses were increased by 56.6% for cases that were initially indeterminate and changes in treatment recommendations occurred in 49.1% of cases. Treatment recommendations were changed to align with the test result in 76.6% of diagnostically challenging cases.

The MDS impacts diagnosis and treatment recommendations by dermatopathologists confronted with diagnostically challenging melanocytic lesions. Increased data are needed in order to completely understand how use of the MDS will translate from dermatopathology to clinical practice.

## 1 Introduction

The lifetime risk of someone living in the United States to develop malignant melanoma now stands at approximately 1 in 50 and, with an annual estimated incidence of 76,000, melanoma is the seventh most common cancer among men and women.^[1]^ While malignant melanoma is the most fatal form of skin cancer, many cases are curable if detected early. Approximately 90% of patients with early-stage melanomas are alive and well 10 years later. For those with advanced-stage disease, however, 10-year survival is only 10% to 15%.^[2]^ Early and accurate diagnosis is critical.

Currently, histopathologic evaluation by a dermatopathologist is considered the “gold standard” for the diagnosis of melanocytic lesions. While many melanocytic lesions are accurately diagnosed by conventional light microscopy and a skilled histopathologist, evidence suggests as many as 8% to 20% of lesions are considered ambiguous by pathologists, meaning difficulty exists in definitively and confidently distinguishing the lesion as benign or malignant.^[3–5]^ Factors contributing to this ambiguity include interobserver variability between pathologists, conflicting morphologic features within the lesion, and the complexity of molecular pathways contributing to neoplasia.^[3,6–8]^

To address the diagnostic problems associated with ambiguous melanocytic lesions, more sensitive and objective methods have been sought for distinguishing melanoma from nevi, including immunohistochemistry, array comparative hybridization, fluorescent in situ hybridization, and quantitative measurement of biomarker genes.^[9–13]^ Recently, an adjunctive diagnostic test using quantitative reverse transcription polymerase chain reaction (qRT-PCR) was developed to aid pathologists in objectively assessing melanocytic lesions.^[14]^ This test uses formalin fixed, paraffin-embedded tissue sections, and measures the expression of 23 genes, including genes involved in cell differentiation and immune signaling. A weighted algorithm is applied to the expression levels to produce a melanoma diagnostic score (MDS) capable of differentiating malignant melanoma from benign nevi with a sensitivity of 90% (95% CI of 85–93%) and a specificity of 91% (95% CI of 87–95%).^[14]^

Comprehensive assessment of the value added through the clinical use of these adjunctive molecular tools requires an understanding of the way in which the test results are impacting decision-making by ordering physicians. Earlier studies have demonstrated that use of a molecular diagnostic in the evaluation of ambiguous melanocytic lesions can support a more definitive diagnosis of benign or malignant.^[15]^ The present study aimed to assess the relative influence of the 23-gene MDS on diagnostic decision-making and treatment recommendations among dermatopathologists prospectively submitting melanocytic lesions to a clinical laboratory for melanoma gene expression testing.

## 2 Methods

Representative sections of melanocytic lesions were submitted by US-based dermatopathologists to Myriad Genetic Laboratories, Inc. (Salt Lake City, UT) between May 2014 and August 2014 for clinically validated, diagnostic gene expression testing. Cases meeting the following eligibility criteria were included in a retrospective analysis of data queried from a commercial laboratory database: a completed test requisition form, a clinically valid MDS, and completed pre- and post-test clinical utility surveys. All patient and physician identifiers were removed before analysis and the study protocol was determined to meet criteria for a waiver of consent and waiver of authorization by the Western Institutional Review Board (Puyallap, WA) on February 5, 2014.

Each lesion was analyzed according to the technical specifications of the test.^[16]^ Briefly, representative areas of the melanocytic lesions were macro-dissected from 4 μm thick sections on 5 unstained pathology slides and pooled into a single tube. RNA was extracted from the tissue, cDNA synthesized, and qRT-PCR run to measure the expression of each of 23 genes. A score was calculated on a scale of −16.7 to +11.1 as previously described.^[16]^ Scores from 0 to +11.1 were reported as likely malignant, scores from −16.7 to −2.1 were reported as likely benign, and scores ranging from −2.0 to −0.1 were reported as indeterminate.

Samples were submitted by participating dermatopathologists during the course of normal healthcare operations as part of a prospective clinical experience program. In this program, dermatopathologists submitted for testing any melanocytic lesions they encountered in their clinical practice for which uncertainty existed regarding the histopathologic diagnosis. For each submitted case, the dermatopathologists completed a pre-test survey in which they recorded their favored diagnosis (including histopathologic subtype), their level of confidence in that diagnosis, and what, if any, treatment recommendation they intended to provide at that time. The test was performed and the results were reported to the submitting dermatopathologist, who then completed a post-test survey recording their responses to the same questions presented in the pre-test survey (diagnosis, level of confidence, and treatment recommendations).

Diagnoses were recorded on the surveys as benign, malignant, or indeterminate. Up to 3 histopathologic subtypes were recorded and ranked by likelihood by the submitting dermatopathologist based on the differential diagnosis. The dermatopathologist's diagnostic confidence was recorded using a scale with selections of very unsure, unsure, somewhat unsure, neutral, somewhat confident, confident, and very confident. Choices for treatment recommendation included no further treatment necessary, no further treatment necessary if lesion is completely excised, close clinical surveillance of the biopsy site for possible recurrence, excision with a margin of normal skin, wide local excision, sentinel lymph node biopsy and/or other evaluation for evidence of metastasis, or “Other.”

Within this cohort, a subset of the most diagnostically challenging cases was identified. “Diagnostically challenging” was objectively defined as any ambiguous lesion for which the submitting dermatopathologist indicated a pre-test diagnosis of indeterminate (i.e., neither benign nor malignant could be favored); or indicated a pre-test diagnosis of benign or malignant but recorded a confidence level that was neutral or lower (i.e., very unsure, unsure, somewhat unsure, or neutral).

The sample size of this study was initially set at 220 evaluable tests in order to obtain a lower 95% confidence limit of 5% for change in diagnosis and 10% for change in medical management. Descriptive statistics were calculated for demographic and other baseline characteristics. Counts and proportions were calculated for actual values and changes from pre-test to post-test in diagnosis of the lesion, confidence in the diagnosis, and treatment recommendations. Subtyping was assigned based on the submitting dermatopathologist's highest ranked subtype selection. Subset analyses were performed for subtypes with 30 or more submitted lesions.

In addition, counts and proportions were calculated for upgrade changes and downgrade changes. Upgrade changes included changes to a more invasive treatment recommendation (based on the 6 prespecified choices provided on the clinical utility surveys, with sentinel lymph node biopsy and/or other evaluation for evidence of metastasis being the most invasive and no further treatment necessary being the least invasive). Downgrade changes included changes to a less invasive treatment recommendation. “Other” treatment recommendations were excluded from the computations of upgrade and downgrade changes.

## 3 Results

### 3.1 Baseline characteristics of the melanocytic lesion study cohort

Table 1 summarizes the baseline characteristics of the total population of cases eligible for study inclusion (N = 1695), including age, gender, procedure type, anatomical location of the lesion, diagnosis recorded by the dermatopathologist at time of sample submission, and the MDS and corresponding test result. The most common subtypes were dysplastic nevus (n = 572, 33.7%), melanoma NOS (not otherwise specified) (n = 158, 9.3%), and melanoma in situ other than lentigo maligna (n = 144, 8.5%) (Table 2). Cases were submitted by a total of 79 dermatopathologists.

**Table 1:** Demographic and other baseline characteristics.

**Table 2:** Distribution of tested lesion subtypes.

Of the 1695 cases, 175 (10.3%) were submitted with an indeterminate diagnosis recorded by the dermatopathologist. There were 928 (54.7%) cases submitted with a benign diagnosis and 592 (34.9%) submitted with a malignant diagnosis. A total of 218 (12.9%) patients met the definition of the diagnostically challenging subset. Table 1 provides the baseline characteristics of this diagnostically challenging subset of patients. The most common subtypes in this subset of patients were atypical junctional melanocytic proliferation (n = 44, 20.2%), dysplastic nevus (n = 40, 18.3%), and atypical Spitz tumor (n = 38, 17.4%). All but one atypical Spitz tumor that was submitted for testing was included in the diagnostically challenging subset. These 3 subtypes accounted for 56.0% of all diagnostically challenging cases. The full distribution of subtypes is shown in Table 2.

### 3.2 Impact of the MDS on diagnostic decision-making

Within the subset of diagnostically challenging cases, 175 (80.3%) were submitted with a pre-test diagnosis of indeterminate, 23 (10.6%) with a “favor benign” diagnosis (with low confidence), and 20 (9.2%) with a “favor malignant” diagnosis (with low confidence) (Table 1, Fig. 1). For diagnostically challenging cases initially diagnosed as indeterminate, definitive diagnoses increased by 56.6% following testing. A diagnosis of indeterminate was indicated for 82 cases post-testing, while a definitive diagnosis of benign was indicated in 89 cases and a definitive diagnosis of malignant in 47 cases. Overall, this corresponds to a 42.7% reduction in indeterminate diagnoses. The changes were primarily diagnostic downgrades (from indeterminate to benign), with benign diagnoses increasing 30.2%. Malignant diagnoses increased 12.4% (Table 3, Fig. 1). This reduction in indeterminate diagnoses along with an increase in confidence for benign or malignant diagnoses resulted in an overall decrease in the number of diagnostically challenging cases identified within the total population after testing.

**Figure 1:** Diagnostic changes within difficult to diagnosis melanocytic lesions after review of the MDS. Indeterminate diagnoses were reduced by 42.7% when the MDS became available as part of a comprehensive evaluation of diagnostically challenging cases. Diagnostic changes primarily represented downgrades to a benign diagnosis (30.2%) versus upgrades to a malignant diagnosis (12.4%).

**Table 3:** Change in pre-test and post-test diagnosis.

Similar reductions in indeterminate diagnoses were observed for each of the 3 major subtypes in the diagnostically challenging subset: atypical junctional melanocytic proliferations (43.2%), dysplastic nevi (45.0%), and atypical Spitz tumors (39.5%) (Table 3). The accompanying increases in benign and malignant diagnoses for atypical junctional melanocytic proliferations (25.0% and 18.2%, respectively), dysplastic nevi (30.0% and 15.0%, respectively), and atypical Spitz tumors (31.6% and 7.9%, respectively) were also similar (Table 3).

Among the diagnostically challenging cases that received a benign test result, 5.2% (7/134) had a malignant post-test diagnosis. These cases included superficial spreading melanoma (n = 2) and one each of atypical junctional melanocytic proliferation, atypical Spitz tumor, melanoma, NOS, MELTUMP (melanocytic tumor of uncertain malignant potential), and other (nevus with atypical features). Among the cases that received a malignant test result, 10% (6/60) had a benign post-test diagnosis. These included dysplastic nevus (n = 2) and one each of atypical junctional melanocytic proliferation, atypical Spitz tumor, MELTUMP, and other (cellular nevus).

### 3.3 Impact of the MDS on treatment recommendations

Treatment recommendations were revised in 107 (49.1%) diagnostically challenging cases after the MDS was reported. After excluding 4 “Other” recommendations (2 benign results, 1 malignant result, and 1 indeterminate result) from treatment upgrade and downgrade computations, 79 (76.7%) diagnostically challenging cases that received a modified treatment recommendation were revised in a way that aligned with the test result. For example, 52/132 (39.4%) cases receiving a benign score were downgraded to less invasive recommendations and 27/59 (45.8%) cases receiving a malignant score were upgraded to more invasive recommendations. Conversely, only 13/132 (9.8%) cases receiving a benign score were upgraded to more invasive treatment recommendations and only 5/59 (8.5%) cases receiving a malignant score were downgraded to less invasive recommendations (Table 4, Fig. 2).

**Table 4:** Change in pre-test and post-test treatment recommendations.

**Figure 2:** Changes in treatment recommendations after review of the MDS. Treatment recommendations were revised in 49.1% of diagnostically challenging cases after the MDS was reported to the submitting dermatopathologist. Modifications in treatment recommendations tended to align with the test result, where 39.4% of cases receiving a benign score were downgraded to less invasive recommendations and 45.8% of cases receiving a malignant score were upgraded to more invasive recommendations.

These trends were also observed for the three major subtypes in the subset of diagnostically challenging cases. Overall changes in treatment for atypical junctional melanocytic proliferations (50.0%), dysplastic nevi (60.0%), and atypical Spitz tumors (40.5%) were similar to the overall subset of diagnostically challenging cases. The proportion of treatment recommendations that were changed to align with the test result was also similar for each of the major subtypes relative to all diagnostically challenging cases.

Figure 3 shows an example of an atypical Spitz tumor that was given a final diagnosis of benign nevus after receiving a benign test result. The treatment recommendations were changed from “excision with a margin of normal skin” to “no further treatment necessary if lesion is completely excised.” A case example of a dysplastic nevus that was diagnosed as malignant melanoma after receiving a malignant test result is shown in Fig. 4. In this case, the treatment recommendations were changed from “no further treatment necessary if lesion is completely excised” to “wide local excision.”

**Figure 3:** This lesion from the buttock of a 27-year-old female was submitted as “indeterminate,” with a pre-test differential diagnosis of “atypical Spitz tumor versus Spitz nevus versus Spitzoid melanoma.” The intended pre-test treatment recommendation was “excision with a margin of normal skin.” The MDS was –5.4 (likely benign). A final diagnosis of benign nevus was assigned, and the post-test recommendation was “no further treatment necessary if lesion is completely excised.” Hematoxylin and eosin; original magnification ×20 (A), ×100 (B), ×200 (C), and ×400 (D).

**Figure 4:** This lesion from the left helix of a 53-year-old female was submitted as “indeterminate.” The pre-test differential diagnosis was “dysplastic nevus versus atypical junctional melanocytic proliferation,” and the intended pre-test treatment was “no further treatment necessary if lesion is completely excised” versus “excision with a margin of normal skin.” The MDS was +1.4 (likely malignant). A final diagnosis of malignant melanoma was assigned, and the post-test recommendation was “wide local excision.” Hematoxylin and eosin; original magnification ×20 (A), ×100 (B), ×200 (C), and ×400 (D).

## 4 Discussion

Molecular diagnostics are increasingly utilized to achieve a more objective and reproducible diagnosis of melanocytic lesions.^[8]^ These tests may also support optimized treatment plans based on the adjunctive diagnostic information provided to specific patient cases. Molecular diagnostics are anticipated to offer their maximum clinical utility in ambiguous or diagnostically challenging melanocytic lesions, when the dermatopathologist is unable to confidently provide a definitive diagnosis. The prevalence of diagnostically challenging melanocytic lesions within dermatopathology practice is estimated at 8% to 20%; correspondingly, 12.9% of cases were identified as diagnostically challenging in the present study based upon indeterminate diagnoses or a low level of diagnostic confidence.^[3–5]^

The present study demonstrated within a prospective cohort of diagnostically challenging melanocytic lesions that the MDS impacts diagnoses and treatment recommendations among dermatopathologists. Results show that when the MDS was available to dermatopathologists attempting to distinguish malignant melanoma from benign nevi, definitive diagnoses increased by greater than 50% for those cases that were initially indeterminate and the majority of changes in treatment recommendations were revised to align with the test result. Similar results were observed among the 3 major subtypes included in the diagnostically challenging subset: atypical junctional melanocytic proliferations, dysplastic nevi, and atypical Spitz tumors. Previous studies suggest that the impact of adjunctive diagnostic tests on diagnosis and treatment recommendations may vary based on lesion subtype.^[15]^ However, the findings reported here show that the utility of this gene signature extends to the most common subtypes included in this study.

While the influence of these changes on patient outcomes has not been prospectively quantified, data assessing the sensitivity and specificity of the gene signature in a subset of the retrospective clinical validation cohort has shown that the test accurately classifies melanocytic lesions as benign or malignant in 90% of cases, as compared to available clinical outcomes.^[14,17]^ This suggests that utilizing the MDS in conjunction with histopathology to achieve a more definitive diagnosis in those cases initially considered indeterminate will support an accurate diagnosis that can be used to guide treatment decisions in the majority of cases.

In 9.8% of cases with a benign score and 8.5% of cases with a malignant score, treatment recommendations were changed in a way that was counterintuitive to the test result (upgrades with benign results and downgrades with malignant results). This is not an unexpected result given that the gene expression signature is an adjunctive, rather than absolute, diagnostic tool. It would not necessarily be expected that final diagnoses and treatment recommendations would agree with the score in 100% of cases when the information provided by the test must be considered together with additional clinical and histopathologic features of the case. It is likely that in the limited number of cases where the modified treatment recommendation did not align with the test result the ordering physician observed features independent of the test score that provided greater significance in rendering a final treatment decision than the test result did.

Key stakeholders in the healthcare system, including regulatory agencies, clinical guideline panels, third-party payers, physicians and patients, are increasingly seeking evidence of the clinical utility of diagnostic tests in order to support standard use of such tests in clinical practice.^[18,19]^ While the use of molecular tools in the diagnosis of melanoma is increasing, limited data are available regarding the impact of these techniques in modifying diagnostic evaluations by dermatopathologists.^[8]^ The results of this study demonstrate for the first time in a prospective cohort of diagnostically challenging melanocytic lesions that a novel gene expression signature, and the MDS calculated from it, can impact diagnostic decision-making and treatment recommendations among dermatopathologists. Integration of this test into the pathologic diagnosis of melanocytic lesions has the potential to contribute to more definitive diagnoses and optimized clinical care in the treatment of melanocytic lesions.

## Acknowledgment

We would like to thank Kirstin Roundy for assistance with figure preparation, editing, and formatting the manuscript for submission.
